The article "LncRNA LINC00963 Promotes Tumorigenesis and Radioresistance in Breast Cancer by Sponging miR-324-3p and Inducing ACK1 Expression" was retracted in 2025. Reasons: manipulated images; plagiarized images; overlap with other authors' work; concerns about the images.

# LncRNA LINC00963 Promotes Tumorigenesis and Radioresistance in Breast Cancer by Sponging miR-324-3p and Inducing ACK1 Expression

**DOI:** 10.1016/j.omtn.2019.09.033

**Published:** 2019-10-22

**Authors:** Na Zhang, Xue Zeng, Chaonan Sun, Hong Guo, Tianlu Wang, Linlin Wei, Yaotian Zhang, Jiaming Zhao, Xinchi Ma

**Affiliations:** 1 Department of Radiation Oncology, Cancer Hospital of China Medical University, Liaoning Cancer Hospital & Institute, Shenyang, China

**Keywords:** cell cycle arrest, growth, lncRNA, radioresistance, ROS

## Abstract

Upregulation of long non-coding RNA LINC00963 has been observed in several cancer types. In this study, we analyzed the clinical and biological significance of LINC00963 in breast cancer. The key microRNA (miR) mediating the action of LINC00963 was identified. We show that LINC00963 upregulation is correlated with aggressive parameters of breast cancer. Silencing of LINC00963 suppresses the proliferation and tumorigenesis of breast cancer cells, whereas LINC00963 overexpression exerts an opposite effect. Knockdown of LINC00963 enhances DNA damage and oxidative stress and sensitizes breast cancer cells to radiation. Mechanistically, LINC00963 antagonizes the repressive activity of miR-324-3p on ACK1 expression. Clinically, there is a negative correlation between miR-324-3p and LINC00963 expression in breast cancer tissues. Overexpression of LINC00963 or ACK1 rescues the inhibitory effects of miR-324-3p on breast cancer cell proliferation and radiosensitivity. In addition, knockdown of ACK1 attenuates LINC00963-dependent breast cancer growth and tumorigenesis. Taken together, LINC00963 promotes tumorigenesis and radioresistance in breast cancer through interplay with miR-324-3p and derepression of ACK1. LINC00963 may represent a potential target for the treatment of breast cancer.

## Introduction

Breast cancer is the most common and lethal malignancy in women.^1^ Adjuvant radiotherapy shows benefits in reducing breast cancer recurrence and mortality.^2^^,^^3^ However, the therapeutic efficacy is often hampered by the development of radioresistance in cancer cells.^4^ Understanding the mechanism contributing to radioresistance is pivotal to exploring strategies to improve radiotherapy against breast cancer.

Non-coding RNAs (ncRNAs), which can be classified into small (< 200 nt) and long (> 200 nt) ncRNAs, account for the majority of transcriptomes of a cell.^5^ One class of small ncRNAs, microRNAs (miRNAs) have been found to be involved in a wide range of biological and pathological processes, including development and cancer.^6^ miRNAs bind to the 3′ UTR of target mRNA, leading to repression of mRNA translation or induction of mRNA degradation. Although miRNAs have been well investigated, the role of long ncRNAs (lncRNAs) is poorly determined. Accumulating evidence has established a link between dysregulation of lncRNAs and cancer progression.^7^^,^^8^ For instance, lncRNA AGAP2-AS1 is upregulated in breast cancer and contributes to cancer cell growth and trastuzumab resistance.^9^ lncRNA MIR31HG exerts tumor-suppressive activity in hepatocellular carcinoma through the interplay with miR-575.^10^ Several studies have indicated the implication of lncRNAs in radioresistance of cancer cells.^11^^,^^12^ Zheng et al.^11^ demonstrated that lncRNA SNHG18 upregulation results in radioresistance of glioma cells. Zou et al.^12^ reported that lncRNA OIP5-AS1 is involved in radioresistance of colorectal cancer cells.

The article "LncRNA LINC00963 Promotes Tumorigenesis and Radioresistance in Breast Cancer by Sponging miR-324-3p and Inducing ACK1 Expression" was retracted in 2025. Reasons: manipulated images; plagiarized images; overlap with other authors' work; concerns about the images.

Several lines of evidence have supported an oncogenic role for the lncRNA LINC00963.^13^, ^14^, ^15^, ^16^ Upregulation of LINC00963 has been detected in prostate cancer,^13^ lung cancer,^14^ hepatocellular carcinoma,^15^ and melanoma,^16^ compared to corresponding adjacent noncancerous tissues. Knockdown of LINC00963 was found to suppress prostate cancer cell proliferation, migration, and invasion.^13^ Overexpression of LINC00963 promotes lung cancer cell migration and invasion.^14^ Despite these findings, the expression and function of LINC00963 in breast cancer has not been explored yet.

In this work, we investigated the expression and clinical relevance of LINC00963 in breast cancer. Also, we studied the role of LINC00963 in the regulation of breast cancer cell proliferation, tumorigenesis, and radiosensitivity. In addition, the mechanism involved in LINC00963-dependent aggressive phenotype was clarified.

## Results

### LINC00963 Upregulation Is Associated with Aggressive Features of Breast Cancer

We examined the levels of LINC00963 in 45 paired breast cancer and noncancerous breast tissues by quantitative real-time PCR analysis. The results demonstrated a significant upregulation of LINC00963 in breast cancer specimens in comparison with adjacent noncancerous tissues (p < 0.0001; Figure 1A). Analysis of the relationship between LINC00963 expression and clinicopathologic characteristics (Figure 1B) revealed that elevated LINC00963 expression was significantly associated with tumor size (p = 0.0169) and Tumor, Node, Metastasis (TNM) stage (p = 0.0156). These results suggest an involvement of LINC00963 in breast cancer progression.

**Figure 1:** LINC00963 Upregulation Is Associated with Aggressive Features of Breast Cancer (A) Quantification of LINC00963 levels in 45 paired breast cancer and noncancerous breast tissues by quantitative real-time PCR analysis. (B) Analysis of the relationship between LINC00963 expression and clinicopathological characteristics of patients with breast cancer. (C) Analysis of LINC00963 levels in indicated cell lines. *p < 0.05 versus MCF12A cells.

The article "LncRNA LINC00963 Promotes Tumorigenesis and Radioresistance in Breast Cancer by Sponging miR-324-3p and Inducing ACK1 Expression" was retracted in 2025. Reasons: manipulated images; plagiarized images; overlap with other authors' work; concerns about the images.

### Silencing of LINC00963 Restrains Breast Cancer Proliferation and Tumorigenesis

Compared to MCF12A breast epithelial cells, multiple breast cancer cells (i.e., MDA-MB-231, MCF-7, T47D, and BT474) had an increased expression of LINC00963 (p < 0.05; Figure 1C). To determine the biological function of LINC00963 in breast cancer, we performed knockdown experiments using short hairpin RNA (shRNA) technology in both MCF-7 and MDA-MB-231 cells expressing endogenous LINC00963 at different levels. Transfection with LINC00963-targeting shRNA resulted in significant downregulation of LINC00963 (Figure 2A). Depletion of LINC00963 significantly inhibited the proliferation of MCF-7 and MDA-MB-231 cells, as determined by the 3-(4,5-dimethylthiazol-2-yl)-2,5-diphenyltetrazolium bromide (MTT) (Figure 2B) and 5-Ethynyl-2´-deoxyuridine (EdU) incorporation (Figure 2C) assays. Moreover, knockdown of LINC00963 impaired colony formation in MCF-7 and MDA-MB-231 cells, compared to control cells (p < 0.05; Figure 2D). The effect of LINC00963 knockdown on tumor growth was also examined using a mouse subcutaneous xenograft model. We found that LINC00963-depleted MCF-7 cells developed significantly smaller tumors than control counterparts (p < 0.05; Figure 2E). Consistently, final tumor weight was approximately 50% lower in the LINC00963-depleted group than in the control group (p < 0.05; Figure 2F).

**Figure 2:** LINC00963 Knockdown Restrains Breast Cancer Proliferation and Tumorigenesis (A) Knockdown of LINC00963 in MCF-7 and MDA-MB-231 cells using shRNA technology. shCtrl, control shRNA; shLINC00963, LINC00963-targeting shRNA. (B) Cell proliferation was determined by MTT assay. Cell viability was assessed at indicated time points. (C) EdU incorporation assay. The percentage of EdU-positive cells (green) was quantified. Nuclei was stained with Hoechst 33342 (blue). Scale bar, 100 μm. (D) Colony-formation assay. LINC00963 knockdown suppressed colony formation of MCF-7 and MDA-MB-231 cells. (E and F) Tumorigenic studies using control and LINC00963-depleted MCF-7 cells. (E) Tumor growth curves plotted on basis of tumor volume (n = 4). (F) Final tumor weight was determined at 4 weeks after cell implantation. Inserts are representative images of the xenograft tumors. *p < 0.05 versus shCtrl-transfected cells.

### LINC00963 Knockdown Arrests Cell Cycle at the G0/G1 Phase and Stimulates Apoptosis

Next, we analyzed the impact of knockdown of LINC00963 on cell cycle distribution and apoptosis. Flow cytometric analysis revealed a significant increase in the percentage of the G0/G1-phase cells and decrease in the percentage of the S-phase cells in LINC00963-depleted MCF-7 and MDA-MB-231 cells (Figure 3A). Annexin-V/propidium iodide (PI) double staining further demonstrated that LINC00963 depletion significantly induced apoptotic response in MCF-7 and MDA-MB-231 cells compared to control cells (Figure 3B). Biochemically, the cell cycle regulatory proteins cyclin D1 and CDK6 were markedly reduced and p27 was upregulated when LINC00963 was silenced (Figure 3C). Furthermore, LINC00963 knockdown resulted in increased levels of active caspase-3. These data imply that LINC00963 is involved in breast cancer cell proliferation and survival.

The article "LncRNA LINC00963 Promotes Tumorigenesis and Radioresistance in Breast Cancer by Sponging miR-324-3p and Inducing ACK1 Expression" was retracted in 2025. Reasons: manipulated images; plagiarized images; overlap with other authors' work; concerns about the images.

**Figure 3:** LINC00963 Knockdown Arrests Cell Cycle at the G0/G1 Phase and Stimulates Apoptosis (A) Analysis of cell cycle distribution. MCF-7 and MDA-MB-231 (231) cells were transfected with shCtrl or shLINC00963 (shLINC) and subjected to PI staining before flow cytometry. The table (bottom) shows the percentage of cells in each cell cycle phase. (B) Analysis of apoptosis after Annexin-V/PI double staining. Bar graphs (bottom) represent quantification of apoptosis from three independent experiments. *p < 0.05. (C) Western blot analysis of indicated proteins. Numbers indicate fold change relative to the shCtrl-transfected cells.

### LINC00963 Overexpression Accelerates the Growth and Tumorigenesis of Breast Cancer Cells

To complement the knockdown experiments, we performed LINC00963 overexpression studies in MCF-7 and MDA-MB-231 cells. We noted that ectopic expression of LINC00963 (Figure 4A) led to an enhancement of cell proliferation (Figure 4B) and colony formation (Figure 4C). Furthermore, LINC00963 overexpression increased the percentage of the cells at both the S and G2/M phases and decreased the percentage of the G0/G1-phase cells (Figure 4D). However, overexpression of LINC00963 did not affect spontaneous apoptosis of both MCF-7 and MDA-MB-231 cells (data not shown). *In vivo* studies confirmed that LINC00963 overexpression significantly augmented the growth of MCF-7 xenograft tumors compared to control tumors (p < 0.05; Figure 4E). Final tumor weight was higher in the LINC00963 overexpression group than in the control group (p < 0.05; Figure 4F). Collectively, LINC00963 provides a growth advantage in breast cancer cells.

**Figure 4:** LINC00963 Overexpression Accelerates the Growth and Tumorigenesis of Breast Cancer Cells (A) Overexpression of LINC00963 in MCF-7 cells via transfection with the LINC00963-expressin plasmid. (B) Analysis of cell proliferation by MTT assay. (C) Colony-formation assay in MCF-7 cells transfected with the LINC00963-expressin plasmid or empty vector. (D) Analysis of cell cycle distribution after PI staining. Representative flow cytometric histograms of three independent experiments are shown. (E and F) LINC00963 overexpression promoted the growth of MCF-7 xenograft tumors in nude mice. (E) Tumor growth curves plotted on basis of tumor volume (n = 4). (F) Final tumor weight was determined at 4 weeks after cell implantation. Upper panels are representative images of the xenograft tumors. *p < 0.05 versus vector-transfected cells.

The article "LncRNA LINC00963 Promotes Tumorigenesis and Radioresistance in Breast Cancer by Sponging miR-324-3p and Inducing ACK1 Expression" was retracted in 2025. Reasons: manipulated images; plagiarized images; overlap with other authors' work; concerns about the images.

### Targeting LINC00963 Increases Radiosensitivity of Breast Cancer Cells

Next, we tested whether targeting LINC00963 improves radiosensitivity of breast cancer cells. To this end, we exposed LINC00963-depleted MCF-7 and MDA-MB-231 cells to different doses of radiation and measured clonogenic cell survival. The survival fraction was significantly lower in LINC00963-depleted cells than in control cells after irradiation exposure (p < 0.05; Figure 5A), suggesting an increase in radiosensitivity. To get more insight into the mechanism by which LINC00963 affects radiosensitivity of breast cancer cells, we examined the impact of LINC00963 knockdown on irradiation-induced DNA damage and reactive oxygen species (ROS) generation. We found that irradiation treatment remarkably induced ROS formation (Figure 5B) and DNA damage (Figure 5C) in LINC00963-depleted cells compared to control counterparts. These findings suggest that the knockdown of LINC00963 augments radiosensitivity in breast cancer cells via enhancement of DNA damage and ROS generation.

**Figure 5:** Targeting LINC00963 Increases Radiosensitivity of Breast Cancer Cells (A) Clonogenic survival of MCF-7 and MDA-MB-231 cells transfected with shLINC00963 (shLINC) or shCtrl after exposure to different doses of radiation. *p < 0.05 versus shCtrl-transfected cells. (B) Measurement of ROS levels in transfected cells after 6 Gy radiation. (C) Immunofluorescent staining of γ-H2AX in MCF-7 and MDA-MB-231 cells treated as in (B). The percentage of γ-H2AX-positive cells was quantified. Scale bar, 20 μm. *p < 0.05.

### LINC00963 Antagonizes miR-324-3p to Promote Breast Cancer Growth and Radioresistance

To identify the downstream signaling pathways that mediate the enhanced radiosensitivity upon LINC00963 targeting, we used bioinformatic tools (http://starbase.sysu.edu.cn/panCancer.php) to search for LINC00963-related miRNAs. We tested the effects of nine miRNA candidates (i.e., miR-10a-5p, miR-324-3p, miR-511-3p, miR-532-3p, miR-633a, miR-760, miR-766-5p, miR-769-5p, and miR-1321) on the expression of LINC00963 in breast cancer cells. The results showed that overexpression of miR-324-3p significantly repressed the expression of LINC00963 (Figure S1A). However, the other eight miRs tested did not alter the expression of LINC00963. Moreover, LINC00963 overexpression led to a selective inhibition of miR-324-3p expression (Figure S1B). There was a miR-324-3p response element within LINC00963 (Figure 6A). Most importantly, miR-324-3p expression was inversely correlated with LINC00963 expression in breast cancer specimens (*R* = −0.4309, p = 0.0031; Figure 6B). To further validate the interaction between miR-324-3p and LINC00963, we performed a luciferase reporter assay. As a result, overexpression of miR-324-3p significantly repressed the expression of the wild-type LINC00963 reporter, but not the mutant (Figure 6C). These results suggest that LINC00963 is a direct target of miR-324-3p. Moreover, both miR-324-3p and LINC00963 were detected in Ago2 immunoprecipitates obtained from breast cancer cells (Figure 6D). Taken together, these findings suggest an association of LINC00963 with miR-324-3p in breast cancer.

The article "LncRNA LINC00963 Promotes Tumorigenesis and Radioresistance in Breast Cancer by Sponging miR-324-3p and Inducing ACK1 Expression" was retracted in 2025. Reasons: manipulated images; plagiarized images; overlap with other authors' work; concerns about the images.

**Figure 6:** LINC00963 Associates with miR-324-3p in Breast Cancer Cells (A) Bioinformatic analysis revealed a miR-324-3p response element within LINC00963. (B) miR-324-3p expression was inversely correlated with LINC00963 expression in breast cancer specimens (n = 45). (C) Luciferase reporter assay showed that miR-324-3p had the ability to repress the expression of the wild-type (WT) LINC00963 reporter, but not the mutant (mut). *p < 0.05. N.S., no significance. (D) Quantitative real-time PCR detection of miR-324-3p and LINC00963 in Ago2 immunoprecipitates obtained from MCF-7 and MDA-MB-231 cells. *p < 0.05.

The expression of miR-324-3p was significantly reduced in breast cancer relative to adjacent noncancerous tissues (p = 0.011; Figure 7A). The expression level of miR-324-3p was significantly correlated with tumor size (p < 0.0001) and TNM stage (p = 0.0471) (Figure 7B). Consistently, the level of miR-324-3p was lower in breast cancer cell lines than in MCF12A cells (Figure 7C).

**Figure 7:** LINC00963 Antagonizes miR-324-3p to Promote Breast Cancer Growth and Radioresistance (A) Quantification of miR-324-3p levels in 45 paired breast cancer and noncancerous breast tissues by quantitative real-time PCR analysis. (B) Analysis of the relationship between miR-324-3p expression and clinicopathological characteristics of patients with breast cancer. (C) Analysis of miR-324-3p levels in indicated cell lines. *p < 0.05 versus MCF12A cells. (D) Enforced expression of miR-324-3p in MCF-7 cells after transfection with the miR-324-3p-expressing plasmid. *p < 0.05 versus vector-transfected cells. (E) MCF-7 cells were transfected with indicated constructs and tested for viability at different time points by MTT assay. *p < 0.05. (F) Clonogenic survival of MCF-7 cells transfected with indicated constructs after exposure to different doses of radiation. *p < 0.05 for comparisons between vector and miR-324-3p groups as well as miR-324-3p and miR-324-3p plus LINC00963 groups. (G) Measurement of ROS levels in MCF-7 cells after indicated treatments. *p < 0.05.

The article "LncRNA LINC00963 Promotes Tumorigenesis and Radioresistance in Breast Cancer by Sponging miR-324-3p and Inducing ACK1 Expression" was retracted in 2025. Reasons: manipulated images; plagiarized images; overlap with other authors' work; concerns about the images.

We further showed that enforced expression of miR-324-3p (Figure 7D) led to suppression of cell proliferation (Figure 7E) and enhancement of radiosensitivity (Figure 7F) in MCF-7 cells. In addition, irradiation-induced ROS generation was enhanced when miR-324-3p was overexpressed (Figure 7G). The anti-cancer effects of miR-324-3p were significantly antagonized by co-expression of LINC00963. These data suggest that LINC00963 functions as a sponge for miR-324-3p, thus favoring breast cancer progression.

### miR-324-3p Exerts Tumor-Suppressive Activity by Targeting ACK1

Next, we sought to identify direct target genes of miR-324-3p. Bioinformatic analysis based on the TargetScan platform (http://www.targetscan.org/vert_71/) suggest ACK1 as a potential target of miR-324-3p (Figure 8A). Interestingly, overexpression of miR-324-3p significantly suppressed the endogenous expression of ACK1 protein in MCF-7 and MDA-MB-231 cells (Figure 8B). We also measured the effects of miR-324-3p on multiple potential targets, i.e., DACT1, PDRG1, WNT3A, RAB37, and RND2. However, these genes were not regulated by overexpression of miR-324-3p (Figure S2). Luciferase reporter assay demonstrated that the expression of wild-type *ACK1* 3′ UTR reporter was significantly inhibited by overexpression of miR-324-3p (Figure 8C). However, the mutant form with disruption of the putative miR-324-3p binding site was not affected by miR-324-3p. Functionally, inhibition of cell proliferation (Figure 8D) and enhancement of radiosensitivity (Figure 8E) by miR-324-3p was substantially rescued by co-expression of ACK1. These data indicate that ACK1 serves as a direct target for miR-324-3p in breast cancer.

**Figure 8:** miR-324-3p Exerts Tumor-Suppressive Activity by Targeting ACK1 (A) Bioinformatic analysis proposed that the *ACK1* 3′ UTR harbored a potential target site for miR-324-3p. (B) Western blot analysis of ACK1 protein levels in MCF-7 and MDA-MB-231 cells transfected with the miR-324-3p-expressing plasmid or empty vector. Numbers indicate fold change relative to vector-transfected cells. (C) Luciferase reporter assay showed that miR-324-3p repressed the expression of the wild-type (WT) *ACK1* 3′ UTR reporter, but not the mutant (mut). *p < 0.05. N.S., no significance. (D) MCF-7 cells were transfected with indicated constructs and tested for viability at different time points by MTT assay. *p < 0.05. (E) Clonogenic survival of MCF-7 cells transfected with indicated constructs after exposure to different doses of radiation. *p < 0.05 for comparisons between vector and miR-324-3p groups as well as miR-324-3p and miR-324-3p plus ACK1 groups.

The article "LncRNA LINC00963 Promotes Tumorigenesis and Radioresistance in Breast Cancer by Sponging miR-324-3p and Inducing ACK1 Expression" was retracted in 2025. Reasons: manipulated images; plagiarized images; overlap with other authors' work; concerns about the images.

### Derepression of ACK1 Accounts for LINC00963 Pro-oncogenic Activity

Given the overlapped miR-324-3p binding sites in LINC00963 and *ACK1* 3′ UTR (Figures 6A and 8A), we hypothesized that LINC00963 may protect ACK1 from miR-324-3p-mediated repression. In line with this hypothesis, we demonstrated that overexpression of LINC00963 increased the expression of ACK1, which was reversed by co-expression of miR-324-3p (Figure 9A). We next checked whether ACK1 is involved in the pro-oncogenic activity of LINC00963. To this end, we transfected ACK1-targeting shRNAs to LINC00963-overexpressing MCF-7 cells. Intriguingly, knockdown of ACK1 (Figure 9B) remarkably blocked LINC00963-dependent cell proliferation (Figure 9C) and tumorigenesis (Figure 9D). Taken together, LINC00963 sponges miR-324-3p to upregulate the expression of ACK1, consequently exerting pro-oncogenic effects.

**Figure 9:** Derepression of ACK1 Accounts for LINC00963-Induced Breast Cancer Growth and Tumorigenesis (A) Western blot analysis of ACK1 protein in MCF-7 cells transfected with indicated plasmids. (B) Western blot analysis of ACK1 protein in MCF-7 cells transfected with shCtrl or ACK1-targeting shRNA (shACK1). Numbers indicate fold change relative to the control group. (C) MCF-7 cells were transfected with indicated constructs and tested for viability at different time points by MTT assay. *p < 0.05. (D) MCF-7 cells transfected with indicated constructs were inoculated into nude mice to allow the formation of xenograft tumors. Tumor growth curves plotted on basis of tumor volume (n = 4). Inserts are representative images of the xenograft tumors for each group. *p < 0.05.

## Discussion

In this study, we demonstrate that LINC00963 expression is increased in breast cancer relative to adjacent noncancerous tissues. Furthermore, LINC00963 upregulation is significantly associated with more aggressive parameters of breast cancer. Functionally, knockdown of LINC00963 suppresses the proliferation and tumorigenesis of breast cancer cells, whereas overexpression of LINC00963 exerts an opposite effect. In agreement with the findings in several other cancer types,^13^, ^14^, ^15^, ^16^ we have validated the oncogenic activity of LINC00963 in breast cancer.

The article "LncRNA LINC00963 Promotes Tumorigenesis and Radioresistance in Breast Cancer by Sponging miR-324-3p and Inducing ACK1 Expression" was retracted in 2025. Reasons: manipulated images; plagiarized images; overlap with other authors' work; concerns about the images.

We provide evidence that LINC00963 is capable of modulating cell cycle progression in breast cancer cells. Specially, knockdown of LINC00963 leads to a cell cycle arrest at the G0/G1 phase in breast cancer cells, which may partially explain LINC00963-dependent cell growth and tumorigenesis. At the molecular level, we found that LINC00963 depletion inhibits the expression of cyclin D1 and CDK6 and concomitantly induces the expression of p27. It is well known that p27 acts as a cell cycle repressor.^17^ Induction of p27 can impair cell cycle progression and render cells more susceptible to DNA damage.^18^ Therefore, the growth-suppressive activity of LINC00963 is causally linked to alteration of cell-cycle regulatory proteins. We also showed that knockdown of LINC00963 causes a significant apoptosis in breast cancer cells, which involves the activation of caspase-3. These observations collectively underscore the importance of LINC00963 in breast cancer growth and survival.

A small number of lncRNAs, such as OIP5-AS1, TUG1, and UCA1, have been reported to mediate radioresistance in specific cancer types.^12^^,^^19^^,^^20^ Our data add LINC00963 to the list of regulators of cancer radiosensitivity. We showed that LINC00963 depletion leads to radiosensitization of breast cancer cells. The enhanced response to radiation in LINC00963-depleted cells appears to be the result of increased ROS formation and DNA damage. These findings suggest that LINC00963 protects breast cancer cells from oxidative damage induced by irradiation.

Mechanistically, LINC00963 can interplay with miR-324-3p and antagonize the repressive activity of miR-324-3p on gene expression. We found that there is a negative correlation between LINC00963 and miR-324-3p expression in breast cancer specimens. miR-324-3p shows the ability to repress the expression of LINC00963. Moreover, both LINC00963 and miR-324-3p are enriched in the Ago2-containing protein complex, which plays an important role in miR-mediated gene silencing.^19^ Overexpression of miR-324-3p phenocopies the effects of silencing of LINC00963 on the proliferation, radiosensitivity, and ROS production, suggesting this miR as a tumor suppressor in breast cancer. Similarly, miR-324-3p was reported to exert tumor-suppressive effects on colorectal cancer and nasopharyngeal cancer.^20^^,^^21^ However, in some cancer types, such as gastric cancer,^22^ miR-324-3p was found to promote tumor progression. These findings suggest that miR-324-3p plays a context-dependent role in cancer development. Of note, overexpression of LINC00963 reverts the proliferation defects and radiosensitization induced by miR-324-3p in breast cancer cells. Taken together, these results suggest that LINC00963 acts as a sponge for miR-324-3p.

The article "LncRNA LINC00963 Promotes Tumorigenesis and Radioresistance in Breast Cancer by Sponging miR-324-3p and Inducing ACK1 Expression" was retracted in 2025. Reasons: manipulated images; plagiarized images; overlap with other authors' work; concerns about the images.

Our data further revealed that repression of ACK1 expression accounts for miR-324-3p-mediated tumor-suppressive activity. ACK1 belongs to the family of non-receptor-tyrosine-kinases and functions as a driver of tumor progression.^23^^,^^24^ It has been documented that knockdown of ACK1 suppresses the proliferation and invasion of breast cancer cells.^25^ Although several miRNAs such as miR-7 have been shown to regulate the expression of ACK1,^26^ we here propose a novel miRNA regulator of ACK1. We showed that miR-324-3p can inhibit the expression of ACK1 through interaction with the 3′ UTR of *ACK1* mRNA. Most importantly, overexpression of ACK1 rescues the effects of miR-324-3p on breast cancer cell growth and radiosensitivity. In addition, knockdown of ACK1 attenuates LINC00963-dependent cell growth and tumorigenesis. Therefore, LINC00963 and miR-324-3p converge on the regulation of ACK1 in breast cancer cells, which provides a molecular mechanism for LINC00963-dependent aggressive phenotype. A previous study has documented that LINC00963 promotes the proliferation and invasion of melanoma cells by interacting with miR-608.^16^ Although we focused on the interplay with miR-324-3p, it is likely that other miRNA partners may also contribute to the oncogenic function of LINC00963.

It should be noted that the number of mice per group in tumorigenic studies is relatively small. Ongoing studies are conducted to validate the oncogenic role of LINC00963 in additional breast cancer models.

In conclusion, we show that LINC00963 upregulation contributes to breast cancer growth and radioresistance and that the miR-324-3p/ACK1 axis is engaged in LINC00963-mediated oncogenic activity. These findings suggest that LINC00963 may represent a promising therapeutic target to improve radiotherapy against breast cancer.

## Materials and Methods

### Collection of Tissue Specimens

In this study, we enrolled 45 breast cancer specimens and their corresponding noncancerous tissues from patients who were diagnosed with breast cancer and underwent surgery at the Cancer Hospital of China Medical University (Shenyang, China). Tissue samples were immediately frozen in liquid nitrogen after surgical resection and stored at −80°C until use. Clinicopathological data were retrieved from patient medical records. The median age at diagnosis was 58 years. No patient received any chemotherapy or radiotherapy before surgery. Disease was staged according to the TNM system of the American Joint Committee on Cancer/Union Internationale Contre le Cancer (AJCC/UICC). Tumor size was defined as the maximal diameter of the primary tumor (T1, ≤ 20 cm; T2, 2–5 cm; T3–T4, > 5 cm). Written informed consent was obtained from each patient. The protocol was approved by the Ethical Committee of China Medical University.

The article "LncRNA LINC00963 Promotes Tumorigenesis and Radioresistance in Breast Cancer by Sponging miR-324-3p and Inducing ACK1 Expression" was retracted in 2025. Reasons: manipulated images; plagiarized images; overlap with other authors' work; concerns about the images.

### Cell Lines

MCF12A, MDA-MB-231, MCF-7, T47D, and BT474 cells were obtained from the Institute of Biochemistry and Cell Biology of the Chinese Academy of Sciences (Shanghai, China). The cells were maintained in DMEM (Invitrogen, Grand Island, NY, USA) supplemented with 10% fetal bovine serum (Sigma, St. Louis, MO, USA) in a humidified incubator containing 5% CO_2_.

### RNA Isolation and Quantitative Real-Time PCR Analysis

Total RNA was extracted from tissue samples and cell lines using TRIzol reagent (Invitrogen). After treatment with RNase-free DNase to eliminate genomic DNA, RNA samples were reverse transcribed into cDNA using the Superscript III reverse transcriptase kit (Invitrogen). Quantitative real-time PCR was carried out using the SYBR green RT-PCR kit (TaKaRa, Dalian, China). The PCR primers are as follows: LINC00963, forward, 5′-GCCAAGGAGGGAGTTGTGGCTGC-3′, and reverse, 5′-CTGTTGCCACACCATGCACCACTCC-3′; β-actin, forward, 5′-GTGGACATCCGCAAAGAC-3′, and reverse, 5′-AAAGGGTGTAACGCAACTA-3′. The relative LINC00963 level was calculated after normalization to β-actin using the 2^−ΔΔCt^ method.^27^ For quantification of miR-324-3p, reverse transcription was performed using the MystiCq microRNA cDNA synthesis mix (Sigma). Quantitative real-time PCR was then conducted using the MystiCq microRNA SYBR Green qPCR ReadyMix with universal and miRNA-specific primers (Sigma). The expression of miR-324-3p relative to U6 RNA was calculated.

### Plasmids

LINC00963-, ACK1-, and miR-324-3p-expressing constructs, as well as pcDNA3.1 + empty vector were purchased from Hanyu BioTechnology (Beijing, China). LINC00963-targeting shRNA was synthesized by Hanyu BioTechnology and cloned to pLKO.1 lentiviral vector. ACK1-targeting and nonspecific negative control shRNAs were purchased from Sigma. The pGL3-LINC00963 and pGL3-ACK1-3′ UTR luciferase reporters were prepared by cloning LINC00963 and ACK1-3′ UTR fragments downstream of firefly luciferase coding sequence, respectively. Site-directed mutagenesis was performed using the QuikChange site-directed mutagenesis kit (Stratagene, La Jolla, CA, USA) according to the manufacturer’s protocol. The plasmid constructs were verified by sequencing.

### Cell Transfection

Transfection of the plasmids to breast cancer cells was achieved using Lipofectamine 3000 (Invitrogen), following the manufacturer’s instructions. Stable cell lines were obtained after selection with G418 or puromycin (Sigma).

### Cell Proliferation Assay

Cells were seeded into 96-well plates (4 × 10^3^ cells/well) and cultured for 24, 48, and 72 h. At different time points, cells were incubated with 3-(4,5-dimethylthiazol-2-yl)-2,5-diphenyltetrazolium bromide (5 mg/mL; Sigma) for 4 h at 37°C. The formazan product was dissolved in dimethyl sulfoxide. Absorbance was measured at 570 nm.

The article "LncRNA LINC00963 Promotes Tumorigenesis and Radioresistance in Breast Cancer by Sponging miR-324-3p and Inducing ACK1 Expression" was retracted in 2025. Reasons: manipulated images; plagiarized images; overlap with other authors' work; concerns about the images.

EdU incorporation assay was also employed to determine cell proliferation, which was performed as described previously.^28^ In brief, cells were seeded into 24-well plates at a density of 3 × 10^4^ cells/well. Cells were then incubated with 20 μM of EdU (Beyotime, Haimen, China) for 6 h prior to fixation with ice-cold 4% paraformaldehyde and permeabilization in 1% Triton X-100. After washing, the cells were incubated with the staining solution for 30 min in the dark. Cells were further labeled with 5 μg/mL of Hoechst 33342 (Beyotime) for 1 h at 37°C. EdU-positive cells were counted under a fluorescence microscope.

### Colony-Formation Assay

Colony-formation assay was performed as described previously.^29^ In brief, cells were plated into 6-well plates at a low density (500 cells/well) and cultured for 10–14 days. Colonies were stained with 0.1% crystal violet (Sigma) and counted.

### *In Vivo* Experiments

Six-week-old female nude mice were purchased from Shanghai Laboratory Animal Center, Chinese Academy of Sciences (Shanghai, China) and housed in specific pathogen-free conditions on a 12-h light/dark cycle with free access to food and water. For measurement of tumor growth, stably transfected MCF-7 cells were subcutaneously injected into nude mice (3 × 10^6^ cells/mouse). Each group included four mice. Tumor volume was measured weekly for 4 weeks. After the last measurement, mice were sacrificed and xenograft tumors were resected and weighed. The experiments involving animals were approved by the Animal Care and Use Committee of the China Medical University.

### Cell Cycle and Apoptosis Analysis

Cell cycle and apoptosis analysis was determined as described previously.^30^ For analysis of cell cycle progression, cells were fixed with 70% ethanol and incubated with 1 mg/mL PI staining solution containing RNase A (50 U/mL; Sigma) for 30 min. DNA content was analyzed on a flow cytometer. For apoptosis analysis, cells were fixed and incubated with PI and Annexin-V-fluorescein isothiocynate (FITC) in the dark. Stained cells were analyzed by flow cytometry.

### Western Blot Analysis

Cells were lysated in radio-immunoprecipitation assay buffer (Cell Signaling Technology, Waltham, MA, USA) with a protease inhibitor cocktail (Sigma). Protein concentration was quantified with the Pierce BCA protein assay kit (Thermo Fisher Scientific, Rockford, IL, USA). Lysates were separated by SDS-PAGE and transferred to polyvinylidene difluoride membranes. After blocking with 5% nonfat milk, the membranes were incubated overnight at 4°C with primary antibodies against cyclin D1, CDK6, p27, cleaved caspase-3, ACK1, and glyceraldehyde-3-phosphate dehydrogenase (GAPDH) (all antibodies from Cell Signaling Technology). After washing, the membranes were then probed with horseradish peroxidase-conjugated secondary antibodies for 1 h at room temperature. Signals were visualized using an enhanced chemiluminescence detection kit (Thermo Fisher Scientific).

The article "LncRNA LINC00963 Promotes Tumorigenesis and Radioresistance in Breast Cancer by Sponging miR-324-3p and Inducing ACK1 Expression" was retracted in 2025. Reasons: manipulated images; plagiarized images; overlap with other authors' work; concerns about the images.

### *In Vitro* Irradiation

Cells were seeded into 6-well plates (600 cells/well) and received different doses of irradiation (0, 2, 6, and 10 Gy). The cells were cultured for 14 days to form colonies. After staining with 0.1% crystal violet, colonies were counted. Surviving fraction was estimated based on the ratio of the number of colonies formed to the number of cells seeded.

### Immunofluorescent Staining

DNA damage was evaluated by examination of gamma histone 2AX (γ-H2AX) foci formation.^31^ In brief, cells received 6 Gy irradiation, fixed with 4% paraformaldehyde, and permeabilized with 0.5% Triton X-100. The cells were then blocked with normal goat serum and incubated overnight at 4°C with anti-phospho-γ-H2AX (Cell Signaling Technology). After washing, the cells were probed with Alexa Fluor 488 conjugated-goat anti-rabbit immunoglobulin G (IgG). Nuclei were counterstained with Hoechst 33342. The percentage of γ-H2AX-positive cells was determined under a fluorescent microscope.

### Measurement of ROS

Intracellular ROS production was assessed using the cellular ROS detection assay kit (Abcam, Cambridge, MA, USA) as per the manufacturer’s protocol. In brief, cells were incubated with 20 μM 2',7'-dichlorodihydrofluorescein diacetate (H2DCFDA) at 37°C for 30 min in the dark. Cells were then washed and resuspended in PBS and analyzed using flow cytometry.

### Luciferase Reporter Assay

MDA-MB-231 cells were co-transfected with luciferase reporters together with the miR-324-3p-expressing construct or empty vector. *Renilla* luciferase-encoding plasmid was used to control transfection efficiency. Transfected cells were harvested after 24 h incubation, and luciferase activities were measured using the dual luciferase reporter assay kit (Promega, Madison, WI, USA). The activity of firefly luciferase was normalized to that of *Renilla* luciferase.

### RNA Immunoprecipitation (RIP) Assay

Ago2 RIP assay was performed as described previously.^32^ In brief, MDA-MB-231 cells were lysed in RIP buffer and incubated with magnetic beads conjugated with Ago2 antibody or negative control IgG (Abcam). The precipitated RNAs were recovered and subjected to quantitative real-time PCR analysis.

The article "LncRNA LINC00963 Promotes Tumorigenesis and Radioresistance in Breast Cancer by Sponging miR-324-3p and Inducing ACK1 Expression" was retracted in 2025. Reasons: manipulated images; plagiarized images; overlap with other authors' work; concerns about the images.

### Statistical Analysis

Data are expressed as mean ± SD and were determined by the Student’s t test or one-way ANOVA followed by Tukey’s post hoc test. Associations between LINC00963 expression and clinicopathologic parameters were analyzed by the chi-square test. The correlation between miR-324-3p and LINC00963 expression was determined by Pearson correlation analysis. The results were considered statistically significant if p < 0.05.

## Author Contributions

N.Z. and X.Z. designed the study, completed the statistical analysis, and drafted the manuscript. C.S., H.G., T.W., L.W., Y.Z., J.Z., and X.M. performed experiments and conducted data collection. All authors read and approved the final manuscript.

## Conflicts of Interest

The authors declare no competing interests.

## Supplemental Information

Document S1. Figures S1 and S2

Document S2. Article plus Supplemental Information
